The article "Prediction and Early Warning of Regional Coordinated Development Based on Convolution Neural Network Algorithm" was retracted in 2023. Reasons: unreliable results or conclusions; concerns about the data; concerns about the results or conclusions; concerns about the peer review.

# Prediction and Early Warning of Regional Coordinated Development Based on Convolution Neural Network Algorithm

**DOI:** 10.1155/2021/7143246

**Published:** 2021-06-19

**Authors:** Xue Wen

**Affiliations:** Xinhua College of Ningxia University, Yinchuan 750021, China

## Abstract

In order to respond to the regional coordinated development of the country, it is necessary to put forward a method that can predict and analyze the development trend according to the current development situation. In view of this, the research will carry on the present situation and forecast analysis to the coordinated development of urban agglomeration in Western China. Firstly, the 3E system is used to establish the regional coordination degree evaluation model, and on this basis, the ellipsoid model is introduced for better coordination degree evaluation. In addition, in order to improve the prediction ability of the model, the convolution neural network is used to realize the big data analysis of the model. The results show that the overall coordination degree of the western urban agglomeration is in a weak coordination state in 2015, but the coordination degree of the region will reach 147.35 in 2020. The results show that the overall coordination degree of western urban agglomeration will gradually show a good trend, but the change speed is slow. The above results show that the prediction model in the study has strong practicability, the calculation results can fit the current situation, and the good prediction ability can provide decision-making suggestions for many governments.

## 1. Introduction

The Third Plenary Session of the 16^th^ Central Committee of the Communist Party of China put forward five overall plans, including regional development, which can gradually narrow the gap between the development of various regions and form a new pattern of complementary advantages and coordinated development in the east, the middle, and the west. However, with the energy and environmental crisis brought about by economic development, the economic crisis in regional development is gradually emerging, so how to achieve regional coordinated development and deal with the problems of energy consumption and environmental pollution brought about by development is extremely important [1]. As a result, some studies have proposed the 3E system for the coordinated development of economy, energy, and environment, and governments at all levels in the world are constantly studying the 3E system, which has become a world-class means to deal with the triple crisis of economy, environment, and energy [2]. However, recently, many studies have estimated the current utilization of land and resources by agriculture and animal husbandry [3, 4], and various studies have studied the environmental changes under the utilization of resources [5], while a few studies have used convolution neural network to study various comprehensive factors in regional coordinated development, which makes 3E system play little role in regional coordinated development. In view of this, the convolution neural network big data analysis algorithm will be applied to the regional coordinated development of the 3E system prediction model, so as to solve the problems in the 3E system and achieve better decision support.

Regional coordinated development will be affected by many factors, so in order to make the three areas of energy, economy, and environment in regional sustainable development develop in a more reasonable mode for a long time, a more reasonable decision-making algorithm is needed. In order to ensure the rapid development of the western region, a convolution neural network algorithm will be used to study the triple problems of energy, economy, and environment in regional coordination. First, through the analysis of the regional 3E system subsystems and then building a comprehensive coordination evaluation model of the 3E system, finally, the convolution neural network algorithm is added to the 3E system to realize the problem prediction and early warning in the coordinated development, so as to realize the coordinated and stable development between regions and promote the sustainable development of all regions.

The innovation of this study is mainly reflected in three aspects. First, simplify the huge data problem in the 3E system. Secondly, the idea of geometry is introduced, and the change trajectory of the 3E system is constructed by using an ellipse model. Finally, a convolution neural network is introduced to analyze the coordination prediction of the 3E system. The above three innovative methods can not only ensure the accuracy of the 3E system in the analysis of multiregional coordinated development and improve the calculation speed of the model but also increase the prediction function of the model, which has a good guiding role for sustainable development of various regions.

The second part summarizes the current situation of regional coordinated development, neural network development, and 3E system research. The third part is to analyze the problems in regional development by constructing the overall framework of the 3E system and use the convolution neural network algorithm for prediction analysis. The fourth part is to analyze the practical effect of the 3E system in practice and explore the prediction and early warning ability of the system. The last part is a summary of this study.

## 2. Literature Review

Since the coordinated regional development strategy was put forward in the Third Plenary Session of the 16^th^ CPC Central Committee, scholars have been analyzing the prospects of coordinated regional development and the problems that may appear in the development. Cai and others applied the improved G1 method based on grey correlation degree, coordination degree model based on bull's-eye distance, and grey target contribution algorithm to analyze the coordinated development degree of the innovation ecosystem and determined the key factors affecting the coordinated development of China's innovation ecosystem [6]. Ha and his team evaluated the development status of regional ecological benefits in the Yangtze River Economic Zone based on relaxation measure and data envelopment analysis model and analyzed the spatial distribution characteristics and evolution law of ecological efficiency by using spatial autocorrelation test model and standard deviation ellipse [7]. Cai and other scholars used the spatial analysis method to analyze the spatial-temporal pattern and power of the coupling and coordinated development of new urbanization and agricultural ecological environment in detail [8]. In 2020, Xu's team used the network analysis method to explore the spatial correlation of regional ecological coordinated sustainable development; found that industrial structure, economic development, and geographical proximity have a positive impact on the spatial spillover of regional ecological efficiency; and put forward corresponding policies [9]. Based on 99 typical coastal plain counties in Jiangsu Province, Xiong et al. optimized and regulated regional urban development imbalance from multiple perspectives [10]. Lu and his research team took 14 cities in Gansu Province as an example to establish the corresponding evaluation index system of coordinated development level of tourism system to understand the evolutionary relationship among regional economy, tourism, and ecological environment [11].

Kelley and others developed a machine learning system combined with a convolutional neural network to predict cell type specific epigenetic and transcriptional profiles in large mammalian genomes, with the purpose of effectively predicting gene expression [12]. Ajita and other scholars used the pretrained volume price neural network to predict gender in eye images obtained from the front camera of smartphones [13]. Chung's team used a representative multichannel convolutional neural network (CNN) to predict the fluctuation of the stock index, and the results show that the multichannel convolutional neural network has a strong prediction performance [14]. In medicine, Wu and other scholars have applied the convolution neural network to establish a risk prediction model for type 2 diabetes, so as to reduce the incidence rate of diabetes in China [15]. At the same time, Zhao and others studied the internal operation mechanism of the carbon emissions trading system and its impact on 3E, taking Beijing Tianjin Hebei region as an example [16]. Wang et al. studied the impact of different power production taxes on China's energy, economy, and environment; established a dynamic recursive computable general equilibrium model to analyze this problem; and proposed that the production tax rate of power enterprises should be appropriately increased [17]. In order to improve the comprehensive benefits, Zhang's team proposed a multiobjective sustainability evaluation method of the remanufacturing system based on energy, economy, and environment, The results show that the established quantitative prediction model has high accuracy [18].

To sum up, the research reports on regional coordinated development are increasing, and some scholars constantly try to apply the neural network in practice, but almost no research attempts to apply the prediction performance of convolution neural network to the risk prediction of regional coordinated development. Therefore, in this study, a convolution neural network algorithm will be introduced into the risk prediction of regional coordinated development, in order to achieve the maximum prediction effect of risk in regional coordinated development and realize sustainable development among regions in China [19].

## 3. Materials and Methods

### 3.1. Structure Framework of the Regional 3E System

China's multiregional economy and society are still in the status of unbalanced development, energy production cannot meet the needs of industrial structure and regional development, and the consequence of rapid economic development is that the environment has been seriously damaged. In the long run, the coordinated development of the region will be seriously affected, so in view of this situation, we need three factors in the region to restrict each other, thus forming a unified whole of energy, economy, and environment, which is called 3E system for short [20–22].

In social development, social economy is the premise of development, which determines the height of the superstructure. Environment is not only the basis of development but also the key to ensuring the sustainable development of society. In practice, when people find that energy, economy, and environment interact and need to restrict each other, they will be combined into a whole, collectively referred to as the 3E system. The structural framework is shown in Figure 1.

Figure 1 shows that the 3E system consists of five subsystems, which are the center of the system and interact with other economic subsystems, environmental subsystems, social development subsystems, and policy control subsystems. Among the other four subsystems, the economic subsystem and social development subsystem interact with each other under economic driving force, and the environment subsystem affects each other under the bearing capacity of the environmental system [23]. The policy control subsystem and social development subsystem influence each other under the social support and interact with the environment subsystem through the policy control. And in all subsystems, we need to use policy control to regulate the macrorelationship between the systems. On this basis, five subsystems in the 3E system restrict and connect each other, so as to help the 3E system realize regional sustainable development [24, 25].

### 3.2. Index Data Optimization of the Regional Coordination 3E System

Regional coordination itself has multi-index uncertainty, and a variety of uncertain information interweaves and influences each other. The economic and environmental differences brought by regional differences make it difficult to quantify the multi-index. Therefore, the establishment of a regional coordination 3E system also needs a set of reasonable index systems for quantitative analysis. The selection of indicators should fully reflect the phased and authenticity of the system, as shown in Figure 2.

As shown in Figure 2, the index selection of the energy subsystem should start from three aspects of energy production, supply, and consumption. As a whole process of energy use, it has obvious periodicity. There are seven economic indicators, namely, national accounts, fixed asset investment, price index, gross output value of the first industry, gross output value of the second industry, gross output value of the third industry, and financial and insurance situation. These seven economic indicators have roughly covered the main content of social economy. For the environmental subsystem, seven indicators are also selected, including forest resources, water resources, urban air quality, wastewater and waste gas discharge and treatment, solid waste treatment and utilization, noise pollution, and domestic waste.

The index data in the 3E system is huge and complex, so it is necessary to reduce the indexes in the system. The reduction algorithm is implemented by MapReduce framework. MapReduce is a strategy to implement parallel tasks, which schedules each branch through the host and monitors the execution of tasks by particles. The execution process is shown in Figure 3.

Figure 3 shows that, in the MapReduce framework, firstly, the input file is divided into pieces, and the data is divided into multiple pieces and assigned to each process fulcrum. Each fulcrum executes the map mapping method in parallel and processes the data through a programming algorithm. Finally, the map classifies the algorithm settlement results and then outputs them to the protocol stage. The reduction method used in the protocol phase takes the output of the previous phase as the input, the new calculation results are obtained by fusion calculation, and the results are stored in the database as output files.

### 3.3. Comprehensive Evaluation of Regional Coordination of the 3E System

The comprehensive evaluation of regional coordination of energy, economy, and environment needs to measure the coordination degree of the three, that is to say, quantitative analysis of the comprehensive development level of the three, and the principal component analysis method is used to determine the evaluation model of regional coordinated development level of the 3E system. Firstly, the index data is dimensionless processed, and the standardized index after processing is shown in the following formula:

(1) $$\begin{array}{c} y_{ij}=\frac{\left(x_{ij}-{\bar{x}}_{j}\right)}{s_{j}}. \end{array}$$

In formula (1), *x*_*ij*_ represents the original index data, while ${\bar{x}}_{j}$ represents the average value of the *j* index, and its value is ${\bar{x}}_{j}=1/m\sum_{j=1}^{m}x_{ij}$. *s* is the standard deviation of the *j* index, and its value is $s_{j}=\sqrt{\left(1/m-1\right)\sum_{j=1}^{m}{\left(x_{ij}-{\bar{x}}_{j}\right)}^{2}}$. Secondly, the correlation coefficient matrix *x*_*ij*_ is calculated as shown in the following equation:

(2) $$\begin{array}{c} r_{ij}=\frac{1}{m-1}y_{ii}y_{ij},\;\left(i,j=1,2,...,n\right). \end{array}$$

The correlation coefficient matrix *x*_*ij*_ in equation (2) represents the correlation coefficients of indexes *i* and *j*, *n* represents the total number of indexes, and *m* represents the degree of freedom. Then, the eigenvalue and eigenvector of *r*_*ij*_ are calculated, as shown in the following equation:

(3) $$\begin{array}{c} R={\left(r_{ij}\right)}_{m\times n}. \end{array}$$

In order to find all the eigenvalues of *R*, let |*λI* − *R*|=0, *λ*1 ≥ *λ*2 ≥ ... ≥ *λn* in the eigenvalues, the unit orthogonal eigenvector *a*=(*a*_1*j*_, *a*_2*j*_, ..., *a*_*nj*_)^*T*^ corresponding to the eigenvalues. The principal component is extracted according to the contribution rate of each principal component, and then the comprehensive score of the subsystem is calculated according to the weight of the principal component factor, as shown in the following equation:

(4) $$\begin{array}{c} u_{i}=\sum_{j=1}^{k}b_{j}F_{j}, \end{array}$$

where *b*_*j*_ represents the weight of each principal component.

In order to improve the accuracy of system calculation of energy, economy, and environment coordination, an ellipsoid model is proposed in the study, which can quantify the geometric model to measure the evolution degree of elements in the system. For the ellipsoid model, the development speed of the subsystem in the 3E system is calculated firstly, as shown in the following formula:

(5) $$\begin{array}{c} \left\{\begin{array}{c} f\left(\text{Ener}\right)=\sum_{i=1}^{l}a_{i}x_{i},i=1,2,\ldots ,l,\\ f\left(\text{Eco}\right)=\sum_{j=1}^{m}b_{j}y_{j},j=1,2,\ldots ,m,\\ f\left(\text{Envi}\right)=\sum_{k=1}^{n}c_{k}z_{k},k=1,2,\ldots ,n, \end{array}\right) \end{array}$$

where *f*(Ener), *f*(Eco), *f*(Envi) represent energy, economy, and environment subsystems; *x*_*i*_, *y*_*j*_, *z*_*k*_ represent indicators in energy, economy, and environment subsystems; *a*, *b*, *c* represent the weight of indicators in energy, economy, and environment subsystems; and *i*, *j*, *k* represent the number of indicators in each subsystem. The premise of determining the development rate is to determine the evolution of the 3E system. The calculation equation is shown as follows:

(6) $$\begin{array}{c} \left\{\begin{array}{c} A=\frac{\text{d}f\left(\text{Ener}\right)}{\text{d}t}=\alpha_{1}f\left(\text{Ener}\right)+\alpha_{2}f\left(\text{Eco}\right)+\alpha_{3}f\left(\text{Envi}\right),\\ B=\frac{\text{d}f\left(\text{Eco}\right)}{\text{d}t}=\beta_{1}f\left(\text{Ener}\right)+\beta_{2}f\left(\text{Eco}\right)+\beta_{3}f\left(\text{Envi}\right),\\ C=\frac{\text{d}f\left(\text{Envi}\right)}{\text{d}t}=\gamma_{1}f\left(\text{Ener}\right)+\gamma_{2}f\left(\text{Eco}\right)+\gamma_{3}f\left(\text{Envi}\right). \end{array}\right) \end{array}$$

In the previous equation, *A* represents the comprehensive development level of energy subsystem after internal and external influence, *B* represents the comprehensive development level of economic subsystem after internal and external influence, *C* represents the comprehensive development level of environmental subsystem after internal and external influence, where *α*, *β*, *γ* indicate the influence degree of each influencing factor. According to the development level of each subsystem, the development speed of the subsystem is calculated, as shown in the following equation:

(7) $$\begin{array}{c} \left\{\begin{array}{c} V_{a}=\frac{\text{d}A}{\text{d}t},\\ V_{b}=\frac{\text{d}B}{\text{d}t},\\ V_{c}=\frac{\text{d}C}{\text{d}t}, \end{array}\right) \end{array}$$

where *V*_*a*_, *V*_*b*_,  and *V*_*c*_ represent the development speed of energy, economy, and environment subsystems, respectively. The coordination degree of the 3E system is calculated by using the comprehensive development speed of the subsystem. The calculation result is shown in the following equation:

(8) $$\begin{array}{c} \left\{\begin{array}{c} \alpha =\arctan\frac{V_{c}}{\sqrt{V_{a}^{2}+V_{b}^{2}}},\\ \beta =\arctan\frac{V_{b}}{\sqrt{V_{a}^{2}+V_{c}^{2}}},\\ \gamma =\arctan\frac{V_{a}}{\sqrt{V_{b}^{2}+V_{c}^{2}}}. \end{array}\right) \end{array}$$

In the previous equation, *α*, *β*, *γ* are the coordination degree of environment and energy economy under the coordination of energy and economic system; the coordination degree of economy and energy economy under the coordination of energy and environmental system; and the coordination degree of energy, economy, and environment under the coordination of the economic and environmental system. The subsystems of the 3E system are inseparable, interact, and constrain each other, so it is necessary to find the comprehensive coordination degree of the three systems, as shown in the following equation:

(9) $$\begin{array}{c} E\left(V_{a},V_{b},V_{c}\right)=\frac{\left(m\left(V_{a},V_{b}\right),m\left(V_{a},V_{c}\right),m\left(V_{b},V_{c}\right)\right)\cdot \left(\alpha ,\beta ,\gamma \right)}{m\left(V_{a},V_{b}\right)+m\left(V_{a},V_{c}\right)+m\left(V_{b},V_{c}\right)}. \end{array}$$

In the previous equation, *α*, *β*, *γ* are, respectively, regarded as the weights of the coordination degree of environment and energy economy, economy and energy economy, energy and economy, and environment. Among them, the judgment standard of coordination degree is when the degree is [20°∼50°]. For quality coordination, [−10°∼20°], [50°∼80°]. For good coordination, [−40°∼−10°], [80°∼110°]. For weak coordination, [−70°∼-40°], [110°∼140°]. Mild discordance [-110°∼−70°], [140°∼180°] is moderate uncoordinated, and [−180°∼−110°] is a serious disharmony.

### 3.4. Prediction Model of Regional Coordinated Development Based on Convolution Neural Network

One of the research focuses is to deeply analyze the coordinated relationship among energy, economy, environment, and other factors in regional coordinated development. Based on the ellipsoid model, this paper introduces the big data analysis method of convolution neural network and establishes the regional coordination degree prediction model of the 3E system. Finally, the prediction model of the 3E system coordination degree based on a convolution neural network is constructed, as shown in Figure 4.

Figure 4 shows that the model first takes the index data of energy, economy, and environment in the regional development as the input, then constructs the big data index system of 3E system, obtains the regional coordination degree samples by using the ellipsoid model, and preprocesses all the data by using the principal component analysis method. Then, the evaluation value and data preprocessing results of regional coordinated development coordination degree are imported into the convolution neural network model for big data analysis, and the data samples are learned and trained. Finally, the coordination degree of regional coordinated development of 3E system can be obtained, and the coordinated development of each region in the future can be predicted and analyzed.

In the prediction model, a convolution neural network algorithm is used to analyze big data. A convolution neural network is a kind of deep feedforward artificial neural network, which has the advantages of accurate extraction of data features and strong classification ability. As a deep learning model, a convolutional neural network mainly includes an input layer, hidden layer, and output layer, as shown in Figure 5.

Figure 5 shows that the hidden layer structure of the convolutional neural network includes a convolution layer, pooling layer, and full connection layer. The input vector is convoluted through the convolution calculation of the convolution layer and then connected with the pooling layer in the way of local connection. Finally, the output is calculated in the full connection layer in the way of full connection and then transferred to the output layer to get the final classification result. In the forward propagation, the calculation method of the eigenvector of the convolution layer input feature of the convolution neural network is shown as follows:

(10) $$\begin{array}{c} X_{j}^{l}=f\left(\sum_{i\in M_{j}}X_{j}^{l-1}*K_{ij}^{l}+b_{j}^{i}\right). \end{array}$$

*X*_*j*_^*l*^ represents the input eigenvector, *K*_*ij*_^*l*^ represents the *j* convolution kernel of the eigenvector, *b*_*j*_^*i*^ represents the corresponding bias parameter in the calculation, and the calculation after the convolution layer is the downsampling calculation of the pooling layer. When *n* eigenvectors are input, the calculation method of the output eigenvector is shown as follows:

(11) $$\begin{array}{c} X_{j}^{l}=f\left(\beta_{j}^{i}\cdot d\left(X_{j}^{l-1}\right)+b_{j}^{i}\right), \end{array}$$

where *f*() denotes the downsampling function and *β*_*j*_^*i*^ and *b*_*j*_^*i*^ denote the bias parameter. The calculation formula of characteristic sampling is as follows:

(12) $$\begin{array}{c} X_{j}^{l}=f\left(\alpha_{j}^{i}\sum_{i\in M_{j}}X_{j}^{l-1}+b_{j}^{i}\right), \end{array}$$

where *α*_*j*_^*i*^ and *b*_*j*_^*i*^ are all expressed as bias parameters in calculation. The calculation formula of the whole connection layer is as follows:

(13) $$\begin{array}{c} X_{j}^{l}=f\left(\sum_{i\in \left(l-1\right)}W_{IJ}\cdot X_{j}^{l-1}+b_{j}^{i}\right), \end{array}$$

where *f*() is the activation function. In the backpropagation, the weight change is calculated layer by layer from the back to the front:

(14) $$\begin{array}{c} \Delta W_{jk}\left(n\right)=\frac{\eta }{1+n}\left(\Delta W_{jk}\left(n-1\right)+1\right)h_{j}\delta_{k}, \end{array}$$

where *W* is the weight of each layer network and *δ* is the parameter variation coefficient of neuron node. Finally, the data is standardized and the result is limited between [0, 1], as follows:

(15) $$\begin{array}{c} \left\{\begin{array}{c} r_{ij}=\frac{x_{ij}-\min\left(x_{ij}\right)}{\max\left(x_{ij}\right)-\min\left(x_{ij}\right)},\\ r_{ij}=\frac{\max\left(x_{ij}\right)-x_{ij}}{\max\left(x_{ij}\right)-\min\left(x_{ij}\right)}. \end{array}\right) \end{array}$$

In the previous equation, the original data is preprocessed by linearization. The first equation preprocesses the larger eigenvalues, and the second equation preprocesses the smaller eigenvalues.

## 4. Results and Discussion

### 4.1. Prediction Efficiency Analysis of the Convolution Neural Network Model

The experiment is based on Windows operating system. The data set is imported for model training and testing. 90% of the data is set as the training set, and the remaining 10% is set as the test set. The prediction efficiency of the CNN model is discussed based on the test accuracy of the CNN model, as shown in Figure 6.

As can be seen from Figure 6(a), the CNN model has the highest accuracy rate in the training set, reaching 0.997, and the KNN model has the lowest. In addition, the CNN model has the highest recall rate, reaching 0.996.  Figure 6(b) shows the comparison of the detection accuracy of the four models in the test set. It can be seen that after the training of the training set, the accuracy of the CNN model is still at the highest level. Although the recall rate of the model is not the highest, the recall rate is close to 0.99, which indicates that the CNN model has high accuracy and high recall rate. As can be seen from Figure 6(c), the KNN model has the fastest detection time in the training set and the test set of the four models, and the cost of improving the speed is that the detection accuracy drops significantly, while the CNN model has the longest detection time. Because the convolutional neural network algorithm needs multilayer computation, the execution efficiency is low, and the detection accuracy of the CNN training set needs to be improved. In addition, the ROC curve is used to analyze the performance of each model, as shown in Figure 7.

It can be seen from Figure 7 that the area under the line of the ROC curve of the four neural network models is far greater than 0.5, indicating that the classification effect of the four models is very good. Comparing the offline area of the ROC curve of the four neural network models, it can be found that the convolution neural network model has a larger offline area, which indicates that the convolution neural network model has the best classification effect.

### 4.2. Empirical Analysis on the Prediction of Coordinated Development of the Regional 3E System

This paper selects the index data of coordinated development of urban agglomeration in Western China as the relevant index data; calculates the development level of energy, economy, and environment of urban agglomeration in Western China by running the principal component analysis method; and finally calculates the coordination degree of 3E system of urban agglomeration in Western China, as shown in Table 1.

It can be seen from Table 1 that the overall coordination degree of the 3E system of western urban agglomeration has gradually changed from the best state in 2010 to a serious uncoordinated state. On this basis, this paper analyzes the coordination degree of each subsystem. It can be found that when there are environmental factors, the degree of coordination is slightly uncoordinated. On the contrary, the coordination degree of energy and economy is always in good condition, and the calculation results of the system are basically consistent with the actual situation. The above results show that the environment of western urban agglomerations has a great impact on the 3E system, and it needs many regional governments to issue corresponding environmental protection policies to promote the long-term development of energy economy and environment. Then, the coordination degree of the 3E system of western urban agglomeration is predicted and analyzed by using the convolution neural network prediction model, and the change trend of regional coordination degree of western urban agglomeration from 2021 to 2035 is shown in Figure 8.

The real line in Figure 8 shows the trend of the actual regional coordination degree, while the dotted line shows the prediction result of the convolution neural network model on the regional coordination degree of the future western urban agglomeration. It can be seen from Figure 8(a) that the coordination degree of the two elements under the constraint of mutual influence remains unchanged in the prediction results. It can be seen from Figure 8(b) that the prediction of coordination degree of the 3E system of western urban agglomeration by convolution neural network shows a small downward trend after 2024 and will remain stable in 2030.

## 5. Conclusion and Policy Implications

Regional coordinated development is one of the important preconditions to promote economic development. This paper analyzes and forecasts the prospect of multiregional coordinated development in China, so as to provide corresponding decision support for the reform and optimization of China's multireal estate industrial structure. Taking the coordinated development of multiregions as the research object, this paper constructs the 3E system of regional coordination. Convolution neural network is introduced into the system, and its big data analysis method is used to predict and analyze the regional coordinated development trend. Through the comparative analysis of different network models, it is verified that the convolution neural network has good prediction performance, and the index data of western urban agglomeration is taken as the research object for empirical analysis. The results show that the coordination degree of the 3E system in western urban agglomeration is improved from 92.77. In 2015, it reached 147.35. In 2020, in the latter prediction model, the prediction results show that the coordination degree of the 3E system of western urban agglomeration gradually begins to slow down, which shows that the big data analysis results show that the government's environmental protection measures will gradually make the regional coordinated development better. The research results of this paper can not only analyze the current development status but also predict the development trend in the next few years. This is of great significance for the state and government to carry out regional coordinated development regulation, which will effectively promote the slow development of China's regional rapid development and also promote the economic development of developed regions.

## Figures and Tables

**Figure 1:** 3E basic structure framework of the system.

**Figure 2:** Index selection of the regional coordination 3E system.

**Figure 3:** MapReduce execution process.

**Figure 4:** Prediction model of regional coordinated development of 3E system based on convolution neural network.

**Figure 5:** Structure diagram of CNN convolutional neural network.

**Figure 6:** Comparison of model test results. (a) Training set. (b) Test set. (c) Comparison of detection time.

**Figure 7:** ROC curves of four neural network models. (a) KNN. (b) XGboost. (c) BPNN. (d) CNN.

**Figure 8:** Prediction results of regional coordination degree of urban agglomeration in Western China. (a) Prediction of coordination degree of the binary system. (b) Coordination degree prediction of the 3E system.

**Table 1:** Coordination degree of regional 3E system in western urban agglomeration.

Particular year	Calculation value of 3E system coordination degree (°)	The actual coordination degree of urban agglomerations in western China
2010	Weak coordination (92.77)	Grudging coordination
2011	Weak coordination (97.49)	Grudging coordination
2012	Weak coordination (103.26)	General maladjustment
2013	Mild discordance (9112.71)	General maladjustment
2014	Mild discordance (119.68)	General maladjustment
2015	Mild discordance (124.71)	Mild maladjustment
2016	Mild discordance (133.29)	Mild maladjustment
2017	Moderate discordance (140.32)	Moderate maladjustment
2018	Moderate discordance (144.91)	Moderate maladjustment
2019	Moderate discordance (149.18)	Moderate maladjustment
2020	Moderate discordance (157.24)	Moderate maladjustment

## Data Availability

The data used to support the findings of this study are available from the corresponding author upon request.
